# TILRR Aggravates Sepsis-Induced Acute Lung Injury by Suppressing the PI3K/Akt Pathway

**DOI:** 10.1155/2022/7341504

**Published:** 2022-08-26

**Authors:** Xiaoyu Wang, Feixue Lin, Lisha Guo

**Affiliations:** ^1^Department of Emergency, Binzhou Medical University Hospital, Binzhou 256600, Shandong, China; ^2^Binzhou Welfare Institute, Binzhou 256600, Shandong, China

## Abstract

Acute lung injury (ALI) is a life-threatening lung change, and 40% of ALI cases result from sepsis. However, the effective treatment for sepsis-induced ALI is limited. It is urgent to explore novel therapeutic targets for ALI caused by sepsis. Anti-inflammatory therapy is a potential effective treatment for sepsis-induced ALI. Toll-like/Interleukin-1 receptor regulator (TILRR) could trigger aberrant inflammatory responses. Nevertheless, the role of TILRR in sepsis-induced ALI remains unknown. Besides, the phosphatidylinositol 3′kinase/protein kinase B (PI3K/Akt) pathway exerts protective effect on sepsis-induced ALI. Thus, the primary aim of the current study was to investigate whether TILRR contributed to sepsis-induced ALI by the PI3K/Akt pathway. To construct the sepsis-induced ALI model, human pulmonary microvascular endothelial cells (HPMVECs) were treated with lipopolysaccharide (LPS). Besides, the mRNA levels and protein levels were determined by quantitative reverse transcription-PCR (qPCR) and Western blot (WB), respectively. Moreover, cell proliferation was identified by the Cell Counting Kit-8 (CCK-8) assay and Annexin V was utilized to detect apoptosis. Furthermore, levels of proinflammatory cytokines and oxidative stress were tested by the enzyme-linked immunosorbent assay (ELISA) while reactive oxygen species (ROS) was determined by the flow cytometer. Results indicated that TILRR was upregulated to suppress the proliferation and induce apoptosis of HPMVECs under LPS treatment. Besides, TILRR induced aberrant inflammatory responses and oxidative stress in HPMVECs under LPS treatment. Mechanistically, TILRR regulated proliferation, apoptosis, inflammatory responses, and oxidative stress in LPS-treated HPMVECs through inactivating the PI3K/Akt pathway. In summary, TILRR aggravated sepsis-induced ALI by suppressing the PI3K/Akt pathway. These results could provide novel therapy targets for sepsis-induced ALI.

## 1. Introduction

ALI is a life-threatening lung change characterized by lung edema formation, alveolar injury, surfactant dysfunction, and neutrophil-derived inflammation [1, 2]. ALI arises from various diseases and pathological conditions including sepsis [1, 3]. Sepsis is one of the leading inducers for ALI, and 40% of ALI cases result from sepsis [4]. However, the effective treatment for sepsis-induced ALI is limited. Thus, it is urgent to explore novel therapeutic targets for sepsis-induced ALI.

Sepsis is induced by the excessive immune response for infections of pathogens [5, 6]. Thus, anti-inflammatory therapy is a potential effective treatment for sepsis-induced ALI [7, 8]. TILRR is a novel identified integral component of innate immune and a critical regulator of genes involved in inflammatory responses [9, 10]. Previous studies have indicated that TILRR could trigger aberrant inflammatory responses. For instance, TILRR induces aberrant inflammatory responses following atherosclerosis-caused myocardial infarction to facilitate the progression of cardiovascular disease [11]. Besides, TILRR enhances the production of proinflammatory cytokines through activating genes related to innate immune responses in cervical epithelial cell [12]. However, the role of TILRR in sepsis-induced ALI remains unknown.

Growing evidence has revealed that the PI3K/Akt pathway exerts protective effect on sepsis-induced ALI. For example, mitochondrial coenzyme *Q* attenuates sepsis-induced ALI by activating the PI3K/Akt pathway [13]. Moreover, HO-1 induction regulated by the PI3K/Akt pathway alleviates sepsis-induced ALI by modulating mitochondrial dynamics [14]. Nevertheless, the effect of TILRR on the PI3K/Akt pathway is largely unclear.

Therefore, the purpose of this study was to investigate whether TILRR contributed to sepsis-induced ALI through regulating the PI3K/Akt pathway, so as to explore potential therapeutic targets for sepsis-induced ALI.

## 2. Materials and Methods

### 2.1. Cell Culture

HPMVECs were obtained from the Cell Bank at the Chinese Academy of Sciences (Shanghai, China). Besides, HPMVECs were cultured with DMEM (Gibco BRL, Grand Island, NY, USA) which contained 10% fetal bovine serum (FBS) (Gibco BRL) in a humidified incubator with 5% CO_2_ at 37°C.

### 2.2. Cell Treatment

To construct the sepsis-induced ALI model, HPMVECs were treated with 1 mg/L LPS (^#^L2630, Sigma-Aldrich, St. Louis, MO, USA) for 24 hours. Besides, HPMVECs were treated with LY294002 (^#^S1105, Selleck Chemicals, Houston, TX, USA) for 24 hours to inhibit the PI3K/Akt pathway. In addition, transfection of TILRR small interfering RNA (siRNA) (siTILRR) and nontargeting siRNA (siNC) into HPMVECs was performed by Lipofectamine 2000 (Thermo Fisher Scientific, Waltham, MA, USA). SiTILRR sequences were synthesized based on published sequences [15].

### 2.3. QPCR

Total RNA from HPMVECs were extracted using the Trizol RNA extraction kit (Tiangen, Beijing, China). Next, 1 *μ*g of RNA was utilized for cDNA synthesis by the PrimeScript II 1st Strand cDNA Synthesis Kit (Takara, Dalian, Liaoning, China). Subsequently, SYBR Premix Ex Taq II (Takara, Dalian, Liaoning, China) was utilized for qPCR analysis performed by the ABI 7000 real-time PCR machine (Applied Biosystems, Foster City, CA, USA). Then, the amount of target RNA was normalized to that of internal control (GAPDH) and the data were analyzed by 2^−△△Ct^ relative to the control sample. The primers used for qPCR were as follows: TILRR forward (5′-ACGGTTGTATACCGGACCGT-3′); TILRR reverse (5′-TAGCACAGTGAGGGCCCGTGTAA-3′); Interleukin-1*β* (IL-1*β*) forward (5′ to −3′); IL-1*β* reverse (5′ to −3′); IL-6 forward (5′ to −3′); IL-6 reverse (5′ to −3′); nuclear factor kappa B (NF-*κ*B) forward (5′ to −3′); NF-*κ*B reverse (5′ to −3′); GAPDH forward (5′-TGGTATCGTGGAAGGACTCATGAC-3′); GAPDH reverse (5′-ATGCCAGTGAGCTTCCCGTTCAGC-3′).

### 2.4. WB

First, RIPA buffer (Cell Signaling Technology, Danvers, MA, USA) was used to isolate proteins from HPMVECs. Then proteins were loaded into SDS-polyacrylamide gel and separated by electrophoresis. Next, proteins were transferred from gel onto the PVDF membrane (Millipore, Bedford, MA, USA) followed by blocking membranes using 5% nonfat milk for 2 hours at room temperature (RT). Subsequently, membranes were incubated with primary antibodies at 4°C overnight and cleaned with tris-buffered saline contained in 0.1% Tween20 (TBST). After cleaning, membranes were incubated with secondary antibodies for 1 hour at RT. Finally, the signals of target proteins were visualized by the chemiluminescence detection kit (Beyotime). The primary antibodies used for WB included TILRR antibody (1 : 1000, ^#^ab105360, Abcam, Cambridge, MA, USA), CDC2 antibody (), p21 antibody (), Akt antibody (), p-AKT antibody (), PI3K antibody (), p-PI3K antibody (), and GAPDH antibody ().

### 2.5. CCK-8 Assay

Briefly, HPMVECs (1 × 10^4^) were seeded into 96-well plates. Next, a volume of 100 *μ*L of medium was supplemented with 10 *μ*L of CCK-8 reagent (Beyotime, Shanghai, China) for 2 hours. Subsequently, OD values were detected at an excitation wavelength of 450 nm to analyze the proliferation level.

### 2.6. Flow Cytometric Analysis for Apoptosis

After indicated transfections, HPMVECs (3 × 10^5^) were collected and suspended in 100 *μ*L of PBS to be incubated with 2 *μ*g/mL of annexin V (Thermo Fisher Scientific) at RT for 15 minutes in the dark. Next, HPMVECs were washed twice with PBS and treated with moderate propidium iodide (PI). Then HPMVECs were analyzed by the FACSARIA flow cytometr (BD Biosciences, San Jose, CA, USA).

### 2.7. Cell Cycle Analysis

HPMVECs (3 × 10^5^) were first digested into the single cell using trypsin (Gibco BRL). Next, HPMVECs were collected by centrifuging at 300 g for 1 minute and fixed with 70% ethanol overnight at −20°C. Then HPMVECs were collected by centrifugation at 500 g for 5 minutes. Subsequently, HPMVECs were incubated with moderate PI in the dark for 30 minutes at 37°C. Finally, stained HPMVECs were analyzed by the FACSARIA flow cytometer (BD Bioscience).

### 2.8. ELISA

The levels of IL-1*β*, IL-6, NF-*κ*B, tumor necrosis factor alpha (TNF-*α*), malondialdehyde (MDA), L-glutathione (GSH), and superoxide dismutase (SOD) were detected by ELISA kits purchased from Solarbio (Beijing, China), according to manufacturer's instruction. Briefly, 10 *μ*L of samples or 50 *μ*L standards in different concentrations were added into the 96-well plate. Triplicates were made for each sample. Except the blank wells, 100 *μ*L of reagent labeled with enzyme was then added into each well to incubate samples or standards at 37°C for 1 hour. After washing by PBS, 50 *μ*L of color reagent A and B were added into each well to incubate samples or standards at 37°C for 15 minutes in the dark. Subsequently, 50 *μ*L of termination solution was added into each well to terminate the reaction. Finally, absorbance at 450 nm was detected by Multiscan MK3 (Thermo Fisher Scientific).

### 2.9. ROS Detection

In this study, intracellular ROS level was identified by the oxidative conversion of 2′, 7′-dichlorodihydrofluorescein diacetate (DCFH-DA) to fluorescent DCF. Briefly, 2 × 10^5^ HPMVECs were incubated with serum-free medium containing 10 *μ*mol/L of DCFH-DA solution (^#^S0033, Beyotime) for 20 min at 37°C. Next, HPMVECs were washed three times with PBS followed by the measurement of DCF fluorescence which was measured using the FACSARIA flow cytometer (BD Bioscience).

### 2.10. Statistical Analysis

In this study, quantitative data of results were present as mean ± standard deviation (SD) followed by analysis of statistical differences utilizing the SPSS software (v20, SPSS Inc., Chicago, IL, USA). Besides, the comparation between the two groups was performed by the unpaired Student's *t*-test, and statistics among multiple groups were carried out using posthoc Tukey's test following one way ANOVA. In addition, *P* < 0.05 was considered as statistically significant in the current study.

## 3. Results

### 3.1. TILRR Is Upregulated to Suppress the Proliferation and Induce Apoptosis of HPMVECs in Sepsis-Induced ALI

To construct the sepsis-induced ALI model, HPMVECs were treated with 1 mg/L of LPS. Next, the expression of TILRR was detected by qPCR and WB. Results showed that LPS increased both the mRNA level and protein level of TILRR in HPMVECs (Figures 1(a) and 1(b)). Besides, silence of TILRR by siRNA reversed the regulatory effect of LPS on TILRR expression while siRNA NC had no effect on TILRR expression (Figure 1(a)).

Subsequently, the proliferation of HPMVECs was detected by CCK8 assay. Results indicated that LPS suppressed the proliferation of HPMVECs, whereas silence of TILRR abolished the inhibitory effect of LPS on the proliferation of HPMVECs (Figure 1(b)). By contrast, LPS induced the apoptosis of HPMVECs while silence of TILRR alleviated the effect of LPS on the apoptosis of HPMVECs (Figure 1(c)). Moreover, LPS inhibited G1/S phase transition and promoted S/G2 phase transition of HPMVECs, and silence of TILRR reversed the effect of LPS on the cell cycle of HPMVECs (Figure 1(d)). Thus, the abovementioned results suggested that TILRR was upregulated to inhibit the proliferation and trigger apoptosis of HPMVECs in sepsis-induced ALI.

### 3.2. TILRR Induces Aberrant Inflammatory Responses and Oxidative Stress in HPMVECs in Sepsis-Induced ALI

Next, the effect of TILRR on inflammatory responses on sepsis-induced ALI was identified. Results found that LPS increased the production of proinflammatory cytokines of HPMVECs including IL-1*β*, IL-6, NF-*κ*B, and TNF*α*, whereas silence of TILRR reversed the effect of LPS on the production of proinflammatory cytokines (Figure 2(a)). These results suggested that TILRR induced aberrant inflammatory responses in sepsis-induced ALI.

Aberrant inflammatory responses usually associate with elevated oxidative stress in ALI [16, 17]. Thus, levels of oxidative stress markers of HPMVECs including MDA and GSH were detected by ELISA. Results revealed that LPS increased levels of MDA and GSH while silence of TILRR abolished the regulatory effect of LPS on levels MDA and GSH (Figure 2(b)). By contrast, LPS reduced the level of oxidative stress inhibitor SOD of HPMVECs and TILRR silence upregulated LPS-reduced SOD level (Figure 2(b)). Therefore, these data suggested that TILRR elevated oxidative stress through inducing aberrant inflammatory responses in sepsis-induced ALI.

### 3.3. TILRR Inhibits the PI3K/Akt Pathway of HPMVECs in Sepsis-Induced ALI

Subsequently, the effect of TILRR on the PI3K/Akt pathway in sepsis-induced ALI was determined. CDC2 and p21 are essential regulators for the cell cycle involved in the PI3K/Akt pathway [18, 19]. WB results showed that LPS downregulated CDC2 protein level, whereas elevated p21 protein level in HPMVECs (Figure 3). Besides, silence of TILRR abolished the regulatory effect of TILRR on CDC2 protein level and p21 protein level in HPMVECs (Figure 3).

Phosphorylation is critical for the activation of PI3K and Akt [20]. Results indicated that LPS decreased phosphorylated PI3K and Akt levels in HPMVECs, whereas silence of TILRR alleviated the effect of LPS on the phosphorylation of PI3K and Akt (Figure 3). Thus, these results suggested that TILRR inhibited the PI3K/Akt pathway of HPMVECs in sepsis-induced ALI.

### 3.4. TILRR Suppresses the Proliferation and Induces Apoptosis of HPMVECs in Sepsis-Induced ALI by the PI3K/Akt Pathway

To identify whether TILRR exerted effects on sepsis-induced ALI through the PI3K/Akt pathway, the inhibitor of PI3K/Akt pathway (LY294002) was utilized. First, the efficiency of LY294002 was determined by WB. Results showed that LPS reduced phosphorylated PI3K and Akt levels in HPMVECs while silence of TILRR alleviated the effect of LPS on the phosphorylation of PI3K and Akt (Figure 4(a)). However, LY294002 decreased TILRR silence-increased phosphorylated PI3K and Akt levels in HPMVECs under LPS treatment (Figure 4(a)).

Subsequently, the proliferation of HPMVECs was further detected. Results revealed that LPS prohibited the proliferation of HPMVECs, yet silence of TILRR attenuated the inhibitory effect of LPS on the proliferation of HPMVECs (Figure 4(b)). Nevertheless, LY294002 abolished the effect of TILRR silence on the proliferation of HPMVECs under LPS treatment (Figure 4(b)). Moreover, LPS triggered the apoptosis of HPMVECs and silence of TILRR alleviated the effect of LPS on the apoptosis of HPMVECs (Figure 4(c)). However, LY294002 reversed the effect of TILRR silence on the apoptosis of HPMVECs under LPS treatment (Figure 4(c)). The above data together suggested that TILRR suppressed the proliferation and induced apoptosis of HPMVECs in sepsis-induced ALI through the PI3K/Akt pathway.

### 3.5. TILRR Induces Aberrant Inflammatory Responses and Oxidative Stress in HPMVECs in Sepsis-Induced ALI by the PI3K/Akt Pathway

Next, we further determine whether TILRR induced aberrant inflammatory responses and oxidative stress in sepsis-induced ALI by the PI3K/Akt pathway. Analysis by qPCR found that LPS increased the mRNA levels of IL-1*β*, IL-6, and NF-*κ*B, whereas silence of TILRR alleviated the effect of LPS on the mRNA expressions of IL-1*β*, IL-6, and NF-*κ*B in HPMVECs (Figure 5(a)). Nevertheless, LY294002 abolished the effect of TILRR silence on the mRNA expressions of IL-1*β* and IL-6 under LPS treatment (Figure 5(a)).

Besides, LPS induced ROS production yet silence of TILRR reversed the effect of LPS on the ROS production in HPMVECs (Figure 5(b)). However, LY294002 abolished the effect of TILRR silence on the ROS production under LPS treatment (Figure 5(b)). Therefore, these results suggested that TILRR triggered aberrant inflammatory responses and oxidative stress in sepsis-induced ALI by the PI3K/Akt pathway.

## 4. Discussion

This study indicated that TILRR was upregulated to suppress the proliferation and induce apoptosis of HPMVECs under LPS treatment. Besides, TILRR induced aberrant inflammatory responses and oxidative stress in HPMVECs under LPS treatment. Mechanistically, TILRR regulated proliferation, apoptosis, inflammatory responses, and oxidative stress in LPS-treated HPMVECs through inactivating the PI3K/Akt pathway.

Growing evidence has indicated that aberrant inflammatory responses usually associate with elevated oxidative stress in ALI. For instance, death-associated protein kinase 1 (Dapk1) stimulates inflammatory responses and oxidative stress through activating p38 map kinase/NF-*κ*B pathway in LPS-induced ALI [16]. Besides, LPS-induced ALI could cause aberrant inflammatory responses and elevated oxidative stress by suppressing the Nrf2 pathway via blocking AMPK phosphorylation [17]. Thus, this study detected the effect of TILRR both on inflammatory responses and oxidative stress in sepsis-induced ALI and found that TILRR caused aberrant inflammatory responses and elevated oxidative stress under septic conditions simultaneously for the first time.

Numerous studies have indicated that aberrant inflammatory responses and elevated oxidative stress lead to apoptosis in sepsis-induced ALI. For example, excessive inflammatory responses and oxidative stress induce apoptosis through upregulating long noncoding RNA (lncRNA) LincRNA-p21 in sepsis-induced ALI [21]. Besides, aberrant inflammatory responses and elevated oxidative stress stimulate apoptosis through increasing NLR family, pyrin domain containing 9B (NLRP9b) expression in murine, and cell models of sepsis-induced ALI [22]. Our results showed that TILRR induced apoptosis of HPMVECs in sepsis-induced ALI, suggesting that aberrant inflammatory responses and elevated oxidative stress resulting from sepsis-induced ALI could trigger apoptosis through upregulating TILRR.

Previous studies have demonstrated that the PI3K/Akt pathway exerts protective effect on sepsis-induced ALI. For instance, MitoQ attenuates sepsis-induced ALI by reducing inflammatory responses and oxidative stress via activating the PI3K/Akt pathway [13]. Besides, fibro growth factor-2 (FGF-2) protects against sepsis-induced ALI through effectively blocking inflammatory responses and oxidative stress via activating the PI3K/Akt pathway [23]. Thus, the PI3K/Akt pathway should exert protective effect on sepsis-induced ALI through preventing inflammatory responses and oxidative stress. Moreover, this study found that TILRR aggravated sepsis-induced ALI by suppressing the PI3K/Akt pathway. All these studies together suggested that TILRR exacerbated sepsis-induced ALI through inhibiting the PI3K/Akt pathway to enhance inflammatory responses and oxidative stress.

TILRR is a novel identified integral component of innate immune and a critical regulator of genes involved in inflammatory responses [9, 10]. Previous studies have indicated that TILRR could trigger aberrant inflammatory responses [11, 12]. Similarly, nucleotide oligomerization domain-like receptors with caspase activation and recruitment domain 3 (NLRC3) is essential for immune responses in ALI, which is upregulated in rats with ventilator-induced ALI [24]. Besides, NLRC3 could prohibit PI3K phosphorylation in pulmonary artery smooth muscle cells [25]. Our results showed that TILRR suppressed phosphorylation of PI3K and AKT in HPMVECs under LPS condition. Therefore, TILRR might inhibit phosphorylation of PI3K and AKT by activating NLRC3 to suppress the PI3K/AKT pathway in sepsis-induced ALI.

However, lack of animal experiments to verify *in vitro* results was the limitation of the current study. *In vivo* experiments would be performed to certify our results in the future study.

## 5. Conclusion

In summary, this study indicated that TILRR exacerbated sepsis-induced ALI by suppressing the PI3K/Akt pathway. These results could provide novel therapy targets for sepsis-induced ALI.

## Figures and Tables

**Figure 1:** TILRR is upregulated to suppress the proliferation and induce apoptosis of HPMVECs in sepsis-induced ALI. (a) The mRNA level and protein level of TILRR in HPMVECs treated with LPS and siTILRR. (b) The proliferation rate of HPMVECs treated with LPS and siTILRR. (c) Representative images of flow cytometric apoptosis assay in HPMVECs treated with LPS and siTILRR. The bar graph indicated the percentage of apoptotic cells in each group. (d) Cell cycle of HPMVECs treated with LPS and siTILRR detected using the flow cytometer. LPS: lipopolysaccharide; siTILRR: TILRR siRNA; siNC: nontargeting siRNA. ^*∗*^*P* < 0.05, ^*∗∗*^*P* < 0.01, and ^*∗∗∗*^*P* < 0.001.

**Figure 2:** TILRR induces aberrant inflammatory responses and oxidative stress in HPMVECs in sepsis-induced ALI. (a) The level of IL-1*β*, IL-6, NF-*κ*B, and TNF*α* in HPMVECs treated with LPS and siTILRR detected by ELISA. (b) The level of MDA, GSH, and SOD in HPMVECs treated with LPS and siTILRR detected by ELISA. LPS: lipopolysaccharide; siTILRR: TILRR siRNA; siNC: nontargeting siRNA. ^*∗*^*P* < 0.05, ^*∗∗*^*P* < 0.01, and ^*∗∗∗*^*P* < 0.001.

**Figure 3:** TILRR inhibits the PI3K/Akt pathway of HPMVECs in sepsis-induced ALI. The protein levels of CDC2, p21, Akt, p-Akt, PI3K, p-PI3K in HPMVECs treated with LPS and siTILRR. LPS: lipopolysaccharide; siTILRR: TILRR siRNA; siNC: nontargeting siRNA. ^*∗∗*^*P* < 0.01, ^*∗∗∗*^*P* < 0.001, and ^*∗∗∗∗*^*P* < 0.0001.

**Figure 4:** TILRR suppresses the proliferation and induces apoptosis of HPMVECs in sepsis-induced ALI through the PI3K/Akt pathway. (a) The protein levels of Akt, p-Akt, PI3K, p-PI3K in HPMVECs treated with LPS, siTILRR, and LY294002. (b) The proliferation rate of HPMVECs treated with LPS, siTILRR, and LY294002. (c) Representative images of flow cytometric apoptosis assay in HPMVECs treated with LPS, siTILRR, and LY294002. The bar graph indicated the percentage of apoptotic cells in each group. LPS: lipopolysaccharide; siTILRR: TILRR siRNA; siNC: nontargeting siRNA; LY: LY294002. ^*∗*^*P* < 0.05, ^*∗∗*^*P* < 0.01, and ^*∗∗∗*^*P* < 0.001.

**Figure 5:** TILRR induces aberrant inflammatory responses and oxidative stress in HPMVECs in sepsis-induced ALI by the PI3K/Akt pathway. (a) The mRNA level of IL-1*β*, IL-6, and NF-*κ*B in HPMVECs treated with LPS, siTILRR, and LY294002. (b) The level of ROS in HPMVECs treated with LPS, siTILRR, and LY294002 detected by the flow cytometer. LPS: lipopolysaccharide; siTILRR: TILRR siRNA; siNC: nontargeting siRNA; LY: LY294002. ^*∗*^*P* < 0.05, ^*∗∗*^*P* < 0.01, and ^*∗∗∗*^*P* < 0.001.

## Data Availability

The data used to support the findings of this study are included within the article.
